# Investigating Polyphenol Nanoformulations for Therapeutic Targets against Diabetes Mellitus

**DOI:** 10.1155/2022/5649156

**Published:** 2022-06-21

**Authors:** Fahadul Islam, Jannatul Fardous Khadija, Md. Rezaul Islam, Sheikh Shohag, Saikat Mitra, Saad Alghamdi, Ahmad O. Babalghith, Abdulrahman Theyab, Mohammad Tauhidur Rahman, Aklima Akter, Abdullah Al Mamun, Fahad A. Alhumaydhi, Talha Bin Emran

**Affiliations:** ^1^Department of Pharmacy, Faculty of Allied Health Sciences, Daffodil International University, Dhaka 1207, Bangladesh; ^2^Department of Biochemistry and Molecular Biology, Faculty of Life Science, Bangabandhu Sheikh Mujibur Rahman Science and Technology University, Gopalganj 8100, Bangladesh; ^3^Department of Pharmacy, Faculty of Pharmacy, University of Dhaka, Dhaka 1000, Bangladesh; ^4^Laboratory Medicine Department, Faculty of Applied Medical Sciences, Umm Al-Qura University, Makkah, Saudi Arabia; ^5^Medical Genetics Department, College of Medicine, Umm Al-Qura University, Makkah, Saudi Arabia; ^6^Deputy Manager of Laboratory & Blood Bank, Security Forces Hospital, Makkah, Saudi Arabia; ^7^Department of Cardiology, Z. U Model Hospital, Feni 3900, Bangladesh; ^8^Molecular Pharmacology Research Center, School of Pharmaceutical Sciences, Wenzhou Medical University, Wenzhou 325035, Zhejiang, China; ^9^Department of Medical Laboratories, College of Applied Medical Sciences, Qassim University, Buraydah 52571, Saudi Arabia; ^10^Department of Pharmacy, BGC Trust University Bangladesh, Chittagong 4381, Bangladesh

## Abstract

Diabetes mellitus (DM) is a fatal metabolic disorder, and its prevalence has escalated in recent decades to a greater extent. Since the incidence and severity of the disease are constantly increasing, plenty of therapeutic approaches are being considered as a promising solution. Many dietary polyphenols have been reported to be effective against diabetes along with its accompanying vascular consequences by targeting multiple therapeutic targets. Additionally, the biocompatibility of these polyphenols raises questions about their use as pharmacological mediators. Nevertheless, the pharmacokinetic and biopharmaceutical properties of these polyphenols limit their clinical benefit as therapeutics. Pharmaceutical industries have attempted to improve compliance and therapeutic effects. However, nanotechnological approaches to overcome the pharmacokinetic and biopharmaceutical barriers associated with polyphenols as antidiabetic medications have been shown to be effective to improve clinical compliance and efficacy. Therefore, this review highlighted a comprehensive and up-to-date assessment of polyphenol nanoformulations in the treatment of diabetes and vascular consequences.

## 1. Introduction

Diabetes mellitus (DM), also known as diabetes, is a metabolic group of disorders and can be characterized by chronic hyperglycemia (high blood sugar levels) [1]. The most prevalent symptoms include increased hunger, thirst, and frequent urination. If left untreated or improperly managed, it can lead to a plethora of complications [2, 3]. While hyperosmolar hyperglycemia, diabetic ketoacidosis, and even mortality are common acute complications of DM, severe chronic problems include cognitive impairment, retinal damage, nerve damage, foot ulcers, and chronic kidney disease [4].

DM is a global burden due to its high morbidity and mortality rates [5]. Around 463 million people are sufferings from DM, estimating to be 700 million by 2045worldwide. According to epidemiological research, diabetes is more common in middle- and low-income countries, with around half of the cases unreported and misdiagnosed [6, 7]. The most common types of diabetes are type 1 diabetes mellitus (T1DM) and type 2 diabetes mellitus (T2DM) (Figure 1). T2DM accounts for 90 to 95% of DM cases, with the remaining 5 to 10% being other types of DM, such as T1DM, gestational diabetes, and other small specialized varieties that are rarely encountered [8]. To minimize the annual death rate from T1DM and T2DM, cost-effective treatment options are being searched substantially [9]. Several antidiabetic drugs are sometimes time-consuming due to not being single-dose treatment regimens; some must be taken for the rest of one's life [10].

Preclinical findings suggested that dietary polyphenols with antidiabetic properties are available in fruits, vegetables, etc. [11]. A comprehensive systematic review found an association between a polyphenol-rich diet intake and reduced risk conditions of diabetes [12, 13]. Polyphenols have also appeared to improve glucose metabolism in clinical studies. For example, regular consumption of apple polyphenols for 12 weeks improved glucose tolerance in adults [14, 15]. Despite the fact that several pathways for antidiabetic properties of polyphenolic compounds have been hypothesized, mostly they are based on in vitro research with pharmaceutical doses, which frequently provide misleading or inconsistent outcomes [16, 17]. However, nanoformulations of polyphenols have been demonstrated to possess the potentiality for delivering naturally prevailing antidiabetic drugs with poor pharmacological properties compared with alternative dosage forms [18]. To improve the therapeutic potential by lowering the frequency of administration, increasing accessibility, and delivering prolonged attributes, the nanodrug delivery method is attracting growing interest in formulation of development studies [19–21].

Therefore, this review aimed to provide a clear-cut explanation of polyphenols and their nanoformulations that are used to treat DM with improved antidiabetic efficacy.

## 2. Bioavailability of Polyphenols

The primary sources of dietary polyphenols include fruits, vegetables, and beverages. Because bioactive components are particularly effective in the prevention of various ailments, it is critical to be aware of their availability. The proportion of nutrients is consumed, absorbed, and metabolized by typical gastrointestinal pathways [22, 23]. Intake of phenolic chemicals in large amounts has little effect on the bioavailability profile [24]. Rein and his colleagues [25] advocated that bioavailability is recognized as the final step in ensuring the bioeffectiveness of phenolic compounds, such as at the dietary level, bioavailability is the proportion of a food that is consumed and digested and therefore a matter of nutritional efficacy. As a result, a number of other factors could obstruct the direct absorption of phenolic compounds found in food. External features include interactions with other molecules, food digestion, and a variety of other intestinal functions [26, 27]. Similarly, bioavailability is affected by a variety of activities, including distribution, liberation, elimination, absorption, and metabolic phases, whereas limiting variables, such as intestinal level absorption, restrict bioavailability [25]. Gallic acid and low molecular weight isoflavones are easily absorbed through the gastrointestinal tract (GIT) [24]. Many phenolic compounds, on the other hand, are absorbed at a rate of 0.30–43% and have a low metabolite level circulating in the plasma [25]. Flavonols such as kaempferol and quercetin, on the other hand, have a variety of physiologic in vivo effects [28]. However, due to low absorption rates, low water solubility, and increased instability in alkaline and neutral environments, the bioavailability of these compounds as potential health-promoting components is limited [29]. Apigenin's pure form is also limited in use due to its low solubility and instability [30]. Metabolic events in the oral cavity start the bioavailability of phenolic compounds found in diets. Mastication, for example, is vital in food preparation because it disrupts food components and releases chemicals. When glycosylated phenolic compounds come into contact with bacteria's glycosidase enzymes, they begin to be processed in the oral cavity [31]. According to the research [32], oral microflora enzymes significantly processed anthocyanin detected in fruit extract high in phenolic components and human saliva. After passing through the stomach, just a few molecules are hydrolyzed, while many polyphenols are not. According to Correa-Betanzo and colleagues [33], the gut microbiota's reaction was connected to the stability and change in these dietary components. To be absorbed, certain phenolic components in the GIT must undergo structural changes. Ex vivo studies have demonstrated that phenolic acid is absorbed in the GIT, such as the jejunum and colon, or at the gastric level [26, 34]. The phenolic compounds are assumed to be absorbed by a passive diffusion process or by gastrointestinal carriers such as P-glycoprotein and SGLT1 cotransporters. These transporters, which are expressed on the cell membrane, carry drugs into the cell interior [35, 36]. Aglycones, for example, can move through epithelial cell membranes via passive diffusion [31]. The colon was the site of the first passage reactions, which allowed prior chemical metabolism and, as a result, encouraged absorption. The portal vein transports these compounds from the colon to the liver, and plasma proteins disperse them throughout the bloodstream [37]. Meanwhile, phenolic chemicals are biotransformed in the liver to make them more polar molecules, which will help with their excretion. Phase I involves oxidation and reduction, as well as hydrolysis events catalyzed by the CYP450 enzymes [35], while phase II enhances the hydrophilicity of the molecules prior to elimination [31, 38].

## 3. Causes and Complications of T1DM and T2DM

T1DM is caused by the death of insulin-producing beta cells in the pancreatic islets (Figure 2), resulting in insulin insufficiency. T1DM can be categorized as either idiopathic or immune-mediated. Most T1DM is caused by immunological mediation, in which a T-cell-mediated autoimmune response results in the death of beta cells and, as a result, insulin [39]. The majority of those who are affected are otherwise healthy, having a normal weight at the time of beginning. Insulin sensitivity and responsiveness are frequently normal, especially in the early phases. Despite the fact that T1DM is typically referred to as “juvenile diabetes” due to its consistent beginning in children, the majority of persons with T1DM are now adults. T1DM may be accompanied by unpredictable, irregularly high blood sugar levels, as well as the risk of serious low blood sugar or diabetic ketoacidosis. T1DM patients with these symptoms account for 1–2% of the people [40]. T1DM is partly inherited, with various genes, including several human leukocyte antigen (HLA) genotypes, influencing the chance of developing the disease. Environmental variables, such as food, stress, or viral infection, may play a role in the beginning of DM in those who have a genetic predisposition. Despite the fact that several viruses have been documented, there is no convincing evidence that they can cause DM in humans [41, 42]. Gliadin (a gluten protein) has been described as a dietary factor in the development of T1DM, albeit the mechanism has not been elucidated, at least not completely [43]. T1DM can strike at any age; a considerable percentage of cases have been discovered in adults. T1DM in adults is known as latent autoimmune diabetes of adults (LADA), and it develops more slowly than T1DM in children [44]. Adults with latent autoimmune diabetes are frequently misdiagnosed as having T2DM at first, owing to their age rather than the cause [45].

T2DM, which accounts for 90 to 95% of all DM cases, is caused by insulin resistance, which may include a relative reduction in insulin production (Figure 3). Insulin receptors are thought to be linked to anomalies in the body's sensitivity to insulin. Cases of DM with recognized faults are divided into two categories. Before developing T2DM, many people with T2DM have clinical signs of diabetes (such as poor glucose tolerance and/or impaired fasting glucose) [46]. Lifestyle medications/changes that improve insulin sensitivity or decrease glucose synthesis in the liver may be able to correct or slow the progression of prediabetes to overt T2DM [47]. T2DM is caused mostly by genetics, as well as lifestyle and environmental factors. Obesity (BMI > 30), urbanization, stress, poor diet, and a lack of physical activity are all variables that contribute to the development of T2DM. Dietary factors, such as sugar-sweetened beverages, have been associated with a greater risk of T2DM. Trans-fats and saturated fats raise hazards, while monounsaturated and polyunsaturated fats lessen risks [48]. Excessive eating of carbohydrate-dense foods such as white rice has been linked to an increased risk of diabetes [49]. In certain people, a lack of or insufficient physical activity can raise their risk of developing diabetes.

## 4. Diabetic Status Influences the Bioavailability of Dietary Polyphenols

Hyperglycemia can affect the bioavailability of small-molecule drugs by affecting absorption, distribution, biotransformation, and excretion. In terms of daily dose, component complexity, and food interaction, the bioavailability of medications and dietary polyphenols differs. Polyphenols in food are poorly absorbed, digested, and eliminated. Only about 5–10% of polyphenols are absorbed, and more than 90% of polyphenols that are digested end up in the colon. Clinical drugs, on the other hand, are typically well absorbed and transported to the tissues they are intended to treat. Hyperglycemia has an impact on glucose, protein, and lipid metabolism. The mechanisms that control these metabolic processes are frequently involved in phytochemical biotransformation as well. As a result, hyperglycemia has an impact on dietary polyphenol bioavailability. *C*_max_ and area under the curve (AUC) of mangiferin, baicalin, wogonoside, and oroxyloside were considerably greater in diabetic mice than in healthy mice [50–52]. Phlorizin bioavailability was significantly improved in T2DM rats [53]. Diabetic rats absorbed significantly higher levels of cynaroside, quercetin, luteolin, isorhamnetin, rutin, and formononetin than normal rats [54]. *C*_max_ values for catechin, epicatechin, quercetin, and resveratrol conjugated metabolites were reduced in Zucker diabetic fatty rats [55]. The bioavailability of methylation flavan-3-ol, resveratrol, and quercetin metabolite was dramatically reduced in Zucker diabetic fatty rats [55]. Furthermore, little progress has been made in hyperglycemia-induced changes in the bioavailability of bioactive phytochemicals. Understanding how hyperglycemia affects the bioavailability of dietary polyphenols will aid in improving the benefits and clinical consequences of these phytochemicals [56].

## 5. Polyphenolic Compounds and Their Properties against T1DM and T2DM

### 5.1. Curcumin

Curcumin (Figure 4), a polyphenol, is derived from the turmeric plant's dried root (*Curcuma longa*). Curcumin contains a wide range of pharmacological effects, the most famous of which are anti-inflammatory and antioxidant capabilities [57, 58]. Hepatic stellate cells (HSCs) are the major players in T1DM- and T2DM-related hepatic fibrogenesis [59], and AGEs activate RAGE gene expression in HSCs, which may stimulate HSC activation [58, 59]. Curcumin oral therapy boosted plasma insulin levels, decreased blood glucose levels, and decreased body weight, according to a study [60]. Curcumin improved glucose/lipid metabolic imbalance and increased insulin resistance in diabetic rats, according to a study [61]. The results could be linked to a decrease in TNF-*α* and free fatty acid in serum [4]. Curcumin has antidiabetic properties in both T1DM and T2DM patients. Curcumin protects pancreatic islets from oxidative stress caused by streptozotocin by scavenging free radicals. Curcumin improved insulin secretion, islet viability, reduced reactive oxygen species (ROS) levels, and decreased nitric oxide (NO) production. Oral curcumin reduced hyperglycemia-induced kidney/liver damage in db/db mice by normalizing mitochondrial activity and decreasing lipid peroxidation and NO production [62].

### 5.2. Resveratrol

Resveratrol (3,4′,5-trihydroxy-stilbene, RES) (Figure 4) is a naturally occurring phytoalexin occurring mostly in grains, fruits, vegetables, dry legumes, and plant-derived beverages such as tea, coffee, and wine. Antiobesity, antidiabetes, anticancer, anti-inflammatory, antioxidative, and cardiovascular-protective actions are mostly just a few of the biological and pharmacological characteristics of RES [63–66]. RES has been shown to have glucose-lowering benefits in both T1DM and T2DM in a vast number of *in vivo* studies. Generally, diabetes treatment focuses on lowering blood glucose levels, improving insulin sensitivity, and preserving pancreatic *β*-cells. All of these functions are covered by the protective effects of RES [67–69]. Moreover, multiple studies offered decent research on the therapeutic application of RES for the alleviation of diabetic problems [70].

### 5.3. Quercetin

Quercetin (Figure 4) is a natural flavonoid with antidiabetic effects [71] and the ability to pass the blood-brain barrier (BBB) [72]. Because the brain is one of the organs impacted by diabetes-induced hyperglycemia, dietary components that provide neuroprotection might help reduce the negative effects of the disease [73, 74]. Researchers discovered that quercetin could significantly improve hyperglycemia and insulin resistance [74]. The underlying mode of action was linked to a decrease in endoplasmic reticulum (ER) stress, oxidative stress, and *β*-cell death in the pancreas. Furthermore, many research studies on the use of quercetin in the treatment of DN have been undertaken. By suppressing TGF-*β*1 and connective tissue growth factor (CTGF) overexpression in the kidneys, quercetin could restore renal function in DN rats. Quercetin had the exact opposite effect on insulin-stimulated glucose transporter type 4 (GLUT4) translocation in both the baseline and insulin-resistant states, according to recent research [75].

### 5.4. Apigenin

Apigenin (Figure 4) is a flavone found in various fruits, vegetables, nuts, onions, oranges, and tea [75]. Although alloxan caused an increase in blood cholesterol, hepatic lipid peroxidation, and a decrease in the activity of cellular antioxidants such as catalase (CAT), superoxide dismutase (SOD), and glutathione (GSH), apigenin treatment of diabetic mice alleviated hyperglycemia and improved antioxidants [76]. Apigenin inhibited parathyroid hormone-related protein-stimulated increases in messenger RNA expression levels of extracellular matrix proteins such as collagen 1A1 and fibronectin, proliferating cell nuclear antigen transforming growth factor *β* (TGF-*β*), and interleukin 6 (IL-6) in human pancreatic stellate cells [77, 78]. In streptozotocin (STZ)-induced diabetic rats, apigenin restores the cellular architecture of essential tissues to normal. Additionally, increased glucose transporter type 4 (GLUT4) translocation in response to apigenin therapy supports increased glucose reduction and *β*-cell preservation efficacy [79, 80].

### 5.5. Baicalein

Baicalein (Figure 4), a flavonoid derived from the roots of *Scutellaria baicalensis* Georgi and the fruits of *Oroxylum indicum* (L.) Benth, has been found to have strong antioxidant properties [81, 82]. Fu et al. [83] used an high-fat diet (HFD) and low dosages of STZ to develop diabetes in mice and then fed them an HFD with 0.25 or 0.5 g baicalein/kg diet. Diabetic mice given baicalein had considerably improved hyperglycemia, according to the researchers. They support screening and preclinical research of hydroxyflavones, particularly those with a better pharmacological profile, as prospective treatments for diabetics and their problems [84]. Baicalein also inhibited nuclear factor kappa B (NF-*κ*B) activation, lowered inducible nitric oxide synthase (iNOS) and TGF-*β*1 expression, and improved the structural alterations in renal tissues [85]. Treatment with baicalein also lowered the levels of advanced glycation end products (AGEs) and tumour necrosis factor-alpha (TNF-*α*), decreased NF-*κ*B activation, and prevented histopathological alterations, according to previous findings [86]. Upregulation of AMP-activated protein kinase (AMPK) and its associated signal pathway was the mechanism of action. AMPK is a master regulator of metabolic balance involving inflammation and oxidative stress.

### 5.6. Luteolin

Lutein (Figure 4) is abundant in celery, parsley, broccoli, onion leaves, and chrysanthemum blooms, among other vegetables and fruits [87]. In 3T3-L1 adipocytes and primary mouse adipose cells, luteolin potentiates insulin action and enhances peroxisome proliferator-activated receptor (PPAR) expression and transcriptional activity, and the expression of PPAR target genes such as adiponectin, leptin, and GLUT4, and a PPAR antagonist inhibits this induction [88]. The decrease in circulation levels of inflammatory mediators such as monocyte chemoattractant protein 1 (MCP-1) and resistin, as well as the increase in adiponectin levels in obese mice, is likely to be managed by luteolin's beneficial effects on metabolic pathways implicated in insulin resistance and DM pathogenesis [89]. In diabetic nephropathy, the mechanism of luteolin's renoprotective property could be associated with increased heme oxygenase 1 (HO-1) expression and antioxidant levels [90]. Inflammation-related endothelial insulin resistance was alleviated by luteolin in an IKKb/IRS-1/Akt/eNOS-dependent pathway [91]. Luteolin enhanced insulin production in uric acid-damaged pancreatic *β*-cells by reducing MafA, which decreases mostly via the NF-*κ*B and iNOS-NO signaling pathway [92].

### 5.7. Morin

*Prunus dulcis* (Mill.) D.A. Webb, fruits, and wine were shown to contain morin, a natural flavonoid and a prominent component of traditional medicinal herbs [93, 94]. Oral treatment of morin (Figure 4) for 30 days alleviated hyperglycemia, glucose intolerance, and insulin resistance in animal models. In diabetic rats treated with the morin, high levels of lipid peroxides were reduced, and antioxidant competence was increased. Following treatment, the lipid and lipoprotein profile in the serum was normalized. TNF-*α* levels were reduced after morin treatment [95]. Morin was reported to alleviate high fructose-induced hepatic SphK1/S1P signaling pathway impairment in rat liver and BRL3A cells, resulting in a decrease in hepatic NF-*κ*B activation with IL-1*β*, IL-6, and TNF-*α* levels [96]. Morin then restored hepatic insulin and leptin sensitivity, followed by a reduction in hyperlipidemia and liver lipid buildup in animal and cell line models [97]. Dietary morin inhibitor of PTP1B acts as an insulin receptor activator and sensitizer, activating metabolic pathways [98]. Therefore, in these metabolic actions, morin may have a wide range of beneficial effects in the prevention and management of diabetes.

### 5.8. Catechin

Green tea contains catechin (Figure 4), a natural nonenzymatic plant antioxidant. Tea can quench thirst, calm the mind, function as a diuretic, and be used to treat coughing, weariness, and light sleep, according to ancient Chinese reports; it also contains anti-inflammatory, detoxifying, and expectorant-like qualities. Catechin has been shown to inhibit inflammatory cytokines and activate AMP-dependent/activated protein kinase [99], protein kinase B (Akt) [100], ERK/JNK-p53, and other signaling pathways to maintain normal mitochondrial respiratory chain operation and exert specific therapeutic effects on diabetes in many studies [101]. Catechin also inhibited glucose-degrading enzymes, which helped to prevent diabetes. Catechin not only has distinct antihyperglycemic and antihyperlipidemic properties, but it also has specialized inhibitory effects on diabetes-related comorbidities, particularly DN [102–105]. Catechin was found to serve an important function in the prevention and management of diabetic cataracts. This compound could lower diabetic rat blood sugar levels, improve the expression of HSP27, MDR 2, and MDR3 mRNA in the lens tissue, and prevent and control diabetic retinal cataracts [106–108]. Thus, catechin could be used to develop medications or auxiliary drugs for the treatment of diabetes. Catechin, in particular, protects DNA and reduces oxidative damage, which is a typical entrance site for diabetes and cancer treatment and has significant medical research value.

### 5.9. Naringenin

Naringin (Figure 4), a flavonoid found in grapefruits and citrus fruits, is a common flavonoid. Its antihyperglycemic, antioxidant, and anti-inflammatory effects are well-known [109]. Several recent studies have shown that naringin can help with T1DM and T2DM, as well as the severity of their related health issues; the mechanism is unknown [109, 110]. *In vitro* studies have shown that naringin prevents cells from being destroyed by high glucose levels. Furthermore, naringin has been shown to have therapeutic effects on diabetic complications in multiple studies [111, 112]. Naringin protected rats with HFD/STZ diabetes from diabetes-induced anemia by increasing adiponectin expression and decreasing pro-inflammatory cytokine production. Naringin significantly improved serum glucose levels and lipid profile in rats with NA/STZ-induced DM [109]. In addition to reducing oxidative stress, the effects could be amplified by increasing glycogen phosphorylase and hepatic G6Pase activities, improving insulin secretion response, and promoting GLUT4 expression, adiponectin, and insulin receptor [109].

## 6. Nanoformulations in Diabetes Treatment

### 6.1. Curcumin

Due to its efficacy against T2DM, curcumin has been utilized in food and medicine in Asia for centuries [113–116]. Due to its low water solubility and gastrointestinal stability, it has limited potential for oral delivery [117–121]. Nanodelivery technologies are a different strategy that can increase the stability of those molecules while also increasing curcumin bioavailability [122–131]. Curcumin-loaded PLGA nanoparticles (NPs) with a particle size of 281 nm have been demonstrated to have a better bioavailability when given orally in a diabetic rat model, delaying cataract formation [132]. The self-nano-emulsifying curcumin delivery system was synthesized, with a particle size of 213 nm, and has been proven to increase diabetic neuropathy protection in male Sprague Dawley rats using oral administration systems [133, 134]. A curcumin-loaded NP was recently discovered to have better bioavailability at lower dosage levels [135] Curcumin-loaded PLGA NP with a particle size of 158 nm was synthesized for oral delivery in another investigation, and it showed improved solubility and bioavailability. Nanoformulated curcumin had a 22-fold improvement in oral bioavailability compared with traditional curcumin [136]. Curcumin nano-micelles with a particle size of 17 nm were also created for oral delivery and demonstrated 2 times increase in bioavailability [137].

### 6.2. Resveratrol

Chemical changes, the addition of bioenhancers, the production of RES prodrugs, and the development of innovative pharmaceutical preparations are all alternatives for addressing RES's pharmacological ineptitude [21, 22, 138]. Nanoencapsulation of RES has been shown to be superior to other methods in terms of stability, bioavailability, selective targeting, and increased therapeutic response [138, 139]. RES-loaded layer-by-layer formulations could be used to deliver RES as a medication [140]. In glucose or STZ-treated *β*-TC cells, multilayered RES nanoliposomes produced by dry film hydration and their PEG-amalgamated (PEGylated) modification have been shown to enhance glycaemic status and insulin level. When compared to pure RES, the preparations had a persistent impact *in vitro* for up to 24 hours [141]. In glucose or STZ-exposed *β*-TC cells, resveratrol-loaded nanocochleates produced similar results [142]. As a result, RES-loaded nanoliposomes, PEGylated RES-loaded nanoliposomes, and RES-loaded nanocochleates may be useful formulations for the treatment of T2DM and its microvascular complications [141, 142]. The formulation of RES-loaded casein NPs was proven to be an excellent strategy for the oral delivery of RES, fast penetration, and prolonged drug release. This formulation has been exhibited to enhance resveratrol oral bioavailability by 10-fold [143]. In diabetic rats, RES-loaded solid lipid NPs were found to increase the therapeutic impact of RES after oral administration. Under normal settings, the formulation is allowed for an initial burst followed by a steady release, improving RES oral bioavailability. The formulation was demonstrated to be more efficient than free RES at reversing insulin resistance in T2DM rat sera [143]. Galactosylated PLGA has also been discovered to be a promising nanocarrier for RES oral delivery to increase bioavailability and therapeutic efficacy [144]. In the retina of diabetic rats, oral treatment with RES-assembled gold nanoparticles (AuNPs) inhibited the activation of vascular endothelial growth factor (VEGF) 1, monocyte chemotactic protein 1 (MCP-1), intercellular adhesion molecule 1 (ICAM-1), extracellular signal-regulated kinase (ERK) 1/2, NF-*κ* B, TNF-*α*, IL-6, and IL-1*β* genes. Therefore, RES-assembled AuNPs could be used to treat diabetic retinopathy [145]. There has yet to be a report on a diabetic human clinical trial with RES nanoformulation.

### 6.3. Quercetin

Quercetin nanofabrication has opened up novel potentialities for enhancing oral bioavailability, target selectivity, therapeutic efficacy, and compliance. The oral bioavailability of quercetin loaded on PLGA NPs was shown to be five times higher than untreated quercetin. This quercetin nanoformulation provided up to 6 days of quercetin release. Quercetin-PLGA NPs were reported to dramatically reverse hyperglycemia and oxidative stress (kidney and pancreas) in diabetic rats at a dose of 150 mg/kg every fifth day, and at a level of 150 mg/kg/day, the efficacy was shown to be higher than that of pure quercetin [146]. In diabetic mice, quercetin nanorods provided effective quercetin distribution with superior pharmacological properties in reversing hyperglycemia, alterations in glucose-metabolizing enzymes, and oxidative stress. Nanorods have been shown to improve diabetes treatment efficiency by increasing cellular absorption and bio-distribution of quercetin in the target areas [147]. In PEG-PLA with quercetin in rats, nanocarriers significantly improved the therapeutic potential of quercetin compared with free quercetin in the control of diabetes and associated nephropathy by increasing quercetin serum content [148]. When compared to native oral quercetin, oral distribution of quercetin-succinylated chitosan-alginate core-shell-corona-shaped NPs significantly enhanced oral hypoglycaemic properties of quercetin in diabetic rats [149]. In the therapy of diabetes in rats, quercetin-loaded Soluplus micelles were reported to enhance oral bioavailability (≥16%) and preserve a sustained release pattern [150]. When compared to free quercetin, oral administration of quercetin-conjugated superparamagnetic iron oxide nanoparticles improved diabetes-induced memory impairment in rats at a substantially lower dose [151]. Several quercetin nanoformulations have been reported to enhance oral bioavailability and therapeutic effects against diabetes; nevertheless, clinical findings on quercetin nanoformulation's antidiabetic potential have yet to be published.

### 6.4. Apigenin

Several nanoformulations have been developed to improve apigenin's medicinal efficacy, which has not only increased bioavailability but also confirmed selective targeting. Microwave-synthesized apigenin-pluronic F127 NPs were reported to boost apigenin dissolution rate and oral absorption by more than threefold when compared to the marketed capsule [151]. Apigenin's stability and bioavailability were increased using a carbon nanopowder-based solid dispersion [152]. Apigenin-loaded nanoliposomes have been shown to prevent cardiac cell death in diabetic cardiomyopathy rats [153].

### 6.5. Baicalin

Baicalin is a new antidiabetic bioactive chemical identified exclusively in scutellaria plants, and it has promising bioactivity against T2DM [154, 155]. These bioactive compounds are quite hydrophobic, which limits their bioavailability and, as a result, their functional activity through oral administration systems [156, 157]. Using a nanostructured lipid carrier (NLC) delivery system, a nano-based delivery technique was recently used to increase bioavailability. It demonstrated stronger antidiabetic action than traditional baicalin, limiting medication dose levels [158]. The bioavailability of a baicalin nanoemulsion delivered orally was also studied. The bioavailability of a baicalin-loaded nanoemulsion was shown to be seven times higher than that of the free suspension, suggesting that it could be effective for a variety of therapies, including T2DM. The storage stability of the baicalin-loaded nanoemulsion was also investigated for 6 months, with the results indicating that a uniform particle size provided improved stability [159]. Baicalin-loaded nanoliposomes with a particle size of 375 nm were found to have better bioavailability in a variety of target organs, such as the kidney, liver, and pancreas, in another study [160].

### 6.6. Luteolin

The oral bioavailability of luteolin has been demonstrated to be improved by luteolin nanoformulation [161, 162]. Luteolin-assembled poly (€-caprolactone)-PLGA-nature oil has been proven to be a decent nanocarrier for boosting luteolin dispersion in water and thereby improving oral bioavailability [162]. Luteolin-loaded solid lipid NPs have been shown to improve luteolin's solubility and hence its therapeutic efficacy [163].

### 6.7. Morin

Morin is a phyto-derived bioflavonoid found in many fruits, vegetables, and herbs, and it has been demonstrated to have numerous antidiabetic and antidiabetic properties [164, 165]. Lipogenesis and inflammation are all potential actions. Morin has also been shown to have a stronger hepatoprotective action in some trials, implying that it can lower hyperlipidemia. Morin also has an insulin-mimetic effect and is generally recognized as a naturally produced antidiabetic drug [98, 166]. Its bioavailability is reduced due to its poor oral solubility, resulting in fewer effects. A greater dosage, on the other hand, may cause toxicity. Novel nanodelivery techniques have been researched to enhance bioavailability by oral delivery to overcome such disadvantages [167–169]. Morin-loaded self-nanoemulsifying nanodelivery devices have recently been designed and investigated for oral bioavailability. The enhanced oral bioavailability of these substances has been linked to increased bioactivity in the treatment of a variety of chronic illnesses [168]. Morin was successfully produced utilizing mixed micelles with a particle size of 90 nm in another method. When compared to native substances, the nanosized morin-loaded mixed micelles demonstrated a 3.6-fold increase in cellular absorption, with a 2.4-fold higher permeability rate, which improves bioavailability in systemic circulation [170]. Morin-loaded solid lipid NPs were tested for their usefulness in oral bioavailability in a different way, indicating that a smaller particle size enhances the permeability of the chemical across an intestinal membrane, resulting in a longer release of the compound. Several successful nanotechnology approaches have been employed to increase morin bioavailability during oral delivery, allowing researchers to investigate its promising chronic illness models such asT2DM and its related conditions [171].

### 6.8. Catechins

Catechin nanoscale formulations have previously been shown to increase catechin stability, gastrointestinal absorption, and bioaccumulation [172–177]. In terms of *α*-glucosidase and *α*-amylase inhibitory activities, catechin-grafted inulin was found to have better antidiabetic potential than free catechins and acarbose [178, 179]. Furthermore, catechin-grafted chitosan NPs outperformed native catechins in terms of antioxidant activity [178]. Epigallocatechin-3-gallate-loaded chitosan-peptide NPs have better cellular absorption and antioxidant capacity than free epigallocatechin-3-gallate [180]. Epigallocatechin gallate-loaded cationic lipid NPs have been shown to have promising benefits in reducing ocular inflammation and oxidative stress, indicating that epigallocatechin-3-gallate is likely helpful in diabetes complications [181]. Furthermore, self-assembled gelatin-epigallocatechin gallate NPs were discovered to significantly reduce ocular angiogenesis by targeting integrin *α*v*β*3 [182]. The effective effects of catechins nanoformulations against diabetes and associated problems were predicted in the aforementioned findings. However, to obtain improved therapeutic management in diabetes, more study is needed to produce a unique catechin nanoformulation.

### 6.9. Naringenin

Naringenin is a flavonoid component found in various citrus fruits and beverages, and it has been demonstrated to have powerful antidiabetic properties in a variety of cellular and animal [183–185]. They are often employed to make innovative beverages due to their higher potential activity in several chronic conditions [186, 187]. A naringenin-based nanoemulsion with a particle size of 50 nm was produced, demonstrating increased naringenin bioavailability by oral delivery. The increased bioavailability of naringenin was most likely owing to its improved solubility in self-emulsion nanodelivery devices, which can help it be used more effectively in therapy [186]. Naringenin-loaded NPs with a mean particle size of 66 nm were created, and they had a better bioavailability when administered orally, resulting in improved hepatoprotective efficacy in rat models [188]. In another work, researchers created naringenin-loaded chitosan nanoparticles with a particle size of 407 nm, which had 70% encapsulation effectiveness and increased antioxidant action in in vitro cell models. Although numerous nanodelivery techniques have been tested for oral bioavailability in a variety of illness models, their potential for T2DM animal models and disorders is still restricted [189].

## 7. Conclusion and Future Perspectives

Long-term treatment is essential in the event of chronic metabolic syndrome, such as diabetes. Patient compliance is thus the most significant factor in the development of pharmacotherapeutic drugs for diabetes control. Antidiabetic polyphenolic compounds have a lot of potential for lowering diabetes and its complications. The biopharmaceutical and pharmacokinetic properties of polyphenols limit their therapeutic usefulness. Many antidiabetic nanoformulations have been developed using polyphenolic compounds and nanocrystals. Furthermore, by overcoming pharmacokinetic and biopharmaceutical limitations, nanoscale formulations of polyphenol antidiabetic drugs have been shown to improve therapeutic outcomes. Therefore, nanoformulation development might be seen as a promising approach for achieving the greatest clinical output of polyphenolic antidiabetic compounds. However, more research is required to build clinically potential therapeutic nanoformulations of polyphenolic antidiabetic compounds for the treatment of diabetes and its complications.

## Figures and Tables

**Figure 1:** Pathological events produce type 1 and type 2 diabetes mellitus. The events that lead to type 1 and type 2 diabetes, as well as accompanying biomarkers, are represented schematically. A mix of constitutional and inherited factors produces type 2 diabetes. These factors favor insulin resistance in the early phases of disease progression, which is accompanied by greater insulin and C-peptide concentrations as a counter-regulatory mechanism. As a result, the pancreatic beta cells may be dysregulated, resulting in decreased glucose tolerance. Type 2 diabetes occurs as a result of beta-cell insufficiency, which is accompanied by insufficiently decreased insulin and C-peptide secretion and plasma concentrations as the situation worsens. On the other hand, type 1 diabetes is thought to be caused by a combination of inherited and environmental factors. The earliest stage of type 1 diabetes progression is a mystery. Activating immune cells is hypothesized to set off an autoimmune response, which involves the production of high-affinity autoantibodies against pancreatic beta-cell antigens. Insulin and C-peptide insufficiency develops after beta-cell loss, eventually leading to type 1 diabetes mellitus.

**Figure 2:** Insulin-secreting cells located in the pancreatic islets of Langerhans. Type 1 (insulin-dependent) diabetes is caused by the immune system recognizing and targeting proteins on the surface of beta cells, possibly mistaking them for proteins on an invading organism. The sequence of events that leads to type 1 diabetes is intricate and poorly understood from there. Insulitis is produced by white blood cells known as cytotoxic or “killer” T cells invading the pancreatic islets and inflaming them. Over the course of years, the beta cells are gradually eliminated. Diabetes symptoms begin to appear after most of them have faded. Researchers seek to learn more about the immune system's attack on beta cells in order to develop techniques to stop the process and prevent or delay the formation of diabetes.

**Figure 3:** Insulin resistance occurs when cells in the muscles, fat, and liver do not respond to insulin properly, preventing glucose absorption from the bloodstream. The pancreas produces more insulin as a result, assisting glucose absorption into the cells.

**Figure 4:** Some polyphenolic compounds that have shown antidiabetic properties.

## Data Availability

All data used to support the findings of this study are included in the article.
